The article "ClusTrack: Feature Extraction and Similarity Measures for Clustering of Genome-Wide Data Sets" was published in 2015. Journal: PLoS One.

# ClusTrack: Feature Extraction and Similarity Measures for Clustering of Genome-Wide Data Sets

**DOI:** 10.1371/journal.pone.0123261

**Published:** 2015-04-16

**Authors:** Halfdan Rydbeck, Geir Kjetil Sandve, Egil Ferkingstad, Boris Simovski, Morten Rye, Eivind Hovig

**Affiliations:** 1 Department of Informatics, University of Oslo, Oslo, Norway; 2 Department of Tumour Biology, The Norwegian Radium Hospital, Oslo University Hospital, Oslo, Norway; 3 Department of Medical Informatics, The Norwegian Radium Hospital, Oslo University Hospital, Oslo, Norway; 4 Statistics For Innovation, Norwegian Computing Center, 0314 Oslo, Norway; 5 Science Institute, University of Iceland, Dunhaga 5, 107 Reykjavik, Iceland; 6 Department of Cancer Research and Molecular Medicine, Norwegian University of Science and Technology, Trondheim, Norway; Scripps Health and The Scripps Research Institute, UNITED STATES

## Abstract

Clustering is a popular technique for explorative analysis of data, as it can reveal subgroupings and similarities between data in an unsupervised manner. While clustering is routinely applied to gene expression data, there is a lack of appropriate general methodology for clustering of sequence-level genomic and epigenomic data, e.g. ChIP-based data. We here introduce a general methodology for clustering data sets of coordinates relative to a genome assembly, i.e. genomic tracks. By defining appropriate feature extraction approaches and similarity measures, we allow biologically meaningful clustering to be performed for genomic tracks using standard clustering algorithms. An implementation of the methodology is provided through a tool, ClusTrack, which allows fine-tuned clustering analyses to be specified through a web-based interface. We apply our methods to the clustering of occupancy of the H3K4me1 histone modification in samples from a range of different cell types. The majority of samples form meaningful subclusters, confirming that the definitions of features and similarity capture biological, rather than technical, variation between the genomic tracks. Input data and results are available, and can be reproduced, through a Galaxy Pages document at http://hyperbrowser.uio.no/hb/u/hb-superuser/p/clustrack. The clustering functionality is available as a Galaxy tool, under the menu option "Specialized analyzis of tracks", and the submenu option "Cluster tracks based on genome level similarity", at the Genomic HyperBrowser server: http://hyperbrowser.uio.no/hb/.

## Introduction

Technological advances, such as high throughput sequencing to map immunoprecipitated chromatin [1], as well as a significant number of other feature mapping techniques of the genome [2, 3], have enabled the collection of genome wide distributional information on genomic features from many organisms, cell types, cell states and functional levels, offering a plethora of analytical possibilities for genomic data on the sequence level [4–6]. A lot of this information is available in the form of genomic tracks—biological features defined relative to coordinates on a defined reference genome [7–9]. Due to the large size of such datasets, and the complex relationships between them, there is a need for exploratory analysis solutions. The unsupervised nature of clustering renders it a powerful tool for hypothesis generation, where any arising hypotheses can be subsequently followed up in more focused analyses, for instance through statistical hypothesis testing of relations between pairs of tracks [8].

The article "ClusTrack: Feature Extraction and Similarity Measures for Clustering of Genome-Wide Data Sets" was published in 2015. Journal: PLoS One.

Cluster analysis is a set of techniques used to group objects. Objects within a group should be more similar to each other than to objects outside the group. There are many algorithms that aim to achieve this general goal. In the present study, we focus on algorithms based on pairwise distances between objects. Feature extraction and the definition of similarity between objects are both crucial components of clustering analysis. These components need to be tailored to each particular application.

Although of seemingly broad usefulness, the application of clustering analysis to genomic tracks is not as straightforward as in many other settings, such as in microarray gene expression analysis [10]. In microarray analyses, the set of measured values for a given gene across samples directly constitutes a suitable feature vector. For clustering of genomic tracks, it is far less obvious what should constitute the suitable feature vectors. It is possible to use the per base-pair information as a feature vector, but this is computationally challenging (e.g. a three billion long feature vectors for human analyses) and would often not correspond to meaningful results, as individual base pairs would be considered fully independent.

Here, we introduce a general approach to clustering analysis of genomic track data. To achieve a biologically meaningful clustering, two general questions should be addressed: 1) How should the feature vector be defined, so that each individual element provides an independent piece of information, and 2) How should similarity be defined, so that it corresponds to a biological notion, rather than more arbitrary technical properties (artifacts) of the genomic tracks.

An open source implementation of the approach is provided by a Galaxy [11] tool called “ClusTrack”, available at the Genomic HyperBrowser web server [12]. We demonstrate the usage of our clustering approach on a set of genomic tracks representing occupancy of histone modifications from a range of cell types. We also provide an example of a more focused follow up study based on the results from the clustering analysis. All tracks used in the examples, as well as a large collection of further tracks, are included with the ClusTrack implementation, and are made available at the URL provided at the end of the abstract.

The article "ClusTrack: Feature Extraction and Similarity Measures for Clustering of Genome-Wide Data Sets" was published in 2015. Journal: PLoS One.

## Materials and Methods

A reference genome may be abstracted as a line-based coordinate system [9, 13]. A genomic track refers to a series of data units positioned on such a line. We here consider tracks in the form of points or segments on such a line, which are the most common types of genomic track data, typically represented in gff- or bed-files. The data can be associated with a broad range of biological features, for instance locations of SNPs, genes, DNA methylation, histone modifications or transcription factor binding. Formally, a genomic track can be considered as a feature vector *V*_*i*_, where *i*, ranging from 1 to *N*, is the position in a genome of length *N*. *V*_*i*_ is one if position *i* is covered by a point/segment, and zero otherwise.

### Feature extraction

The task of feature extraction can be defined as the specification of a function from the raw data associated with an object to a vector of values suitable for computing similarity between objects. As a genomic track can be expressed as a vector, it can be used directly as a feature vector for clustering (i.e. using the identity function for feature extraction). This implies measurement of similarity at the resolution of individual base pairs. While this will be useful in some circumstances, it will often not correspond to a desired notion of similarity. As an example: consider a case in which a first track has a point at position *i*, while a second track has a point at position *i* + 1 (and not vice versa). As dimensions *i* and *i* + 1 would be completely independent in a direct feature vector representation of the tracks, such a situation would not contribute to any similarity between the tracks, although it would in many cases signify biological similarity.

In order to accommodate a notion of similarity for proximal point or segment locations (as in the above mentioned case), one needs in some way to consider the dependency between neighboring base pairs. One way of achieving this, is simply to define a set of bins along the genome, computing an aggregated measure for each such bin. For instance, the number or coverage of points/segments can be counted per gene or per chromosome. Then, the aggregated measures per bin together constitute the feature vector for a given track. Formally, we define bin *j* as a set *k*_*j*_ of consecutive genome positions (*k*_*j*_ = [*q*, *r*], where 1 ≤ *q* ≤ *r* ≤ *N* for a genome of length *N*). The aggregative measure is defined as a function *g*, so that *g*(*V*_*k*_*j*__) gives the aggregate measure on bin *j*. The set *g*(*V*_*k*_1__), *g*(*V*_*k*_2__), … *g*(*V*_*k*_*M*__) then defines a feature vector *F*, corresponding to aggregate measures for *M* bins.

The article "ClusTrack: Feature Extraction and Similarity Measures for Clustering of Genome-Wide Data Sets" was published in 2015. Journal: PLoS One.

The dependency structure between positions does not need to correspond to consecutive positions along the genome. There can be several reasons for this. The set of dependent positions could for instance be located close in the 3D organization of the genome, or they could correspond to locations occupied by a common functional category (e.g. locations covered by genes in the same pathway). A single feature could then correspond to aggregation across an arbitrary set of genome positions, thus generalizing the case of binning described above. Each set of dependent positions may itself be represented as a genomic track (denoted as a reference track—not to be confused with the original set of genomic tracks to be clustered). Aggregating values of a given clustering track across such a reference track thus gives rise to a single feature value for the clustering track. A full feature extraction can then be defined through a set of *M* reference tracks, where aggregation across each reference track will give rise to one out of *M* values of the resulting feature vector. Formally, we define *k*_*j*_ to be a set of (possibly non-contiguous) genome positions covered by a reference track *j* ($k_{j}=\{i;i\in 1\;\ldots \;N,V_{i}^{j}=1\}$). The aggregative measure is as before defined as a function *g* on such a set *k*_*j*_. The feature vector *F* is defined as before.

### Similarity measures

Having defined feature extraction, the next step is how to define similarity of the resulting feature vectors. Formally, what is needed is a function defined on a pair of feature vectors, returning a scalar similarity value. One option is to use standard distance measures, such as the Manhattan or Euclidian distance between a pair of vectors. If the extracted features represent raw measures, such as a plain count of points/segments, technical variation (or artifacts) may easily dominate the measurement of similarity. There are many situations in which a varying total number of genomic elements between tracks simply reflects differences in the availability of data or in the parameterizations of procedures that created the tracks. For instance, the number of integration sites of different viruses may reflect a varying scale of studies for the different viruses, rather than biological distinctions. Therefore, normalized measures per bin are often preferred. One can for example use the proportion of points/segments of a track falling within each bin (or within positions covered by each reference track).

The article "ClusTrack: Feature Extraction and Similarity Measures for Clustering of Genome-Wide Data Sets" was published in 2015. Journal: PLoS One.

In the above discussion, we define similarity through a two-step approach of first normalizing individual feature values and then applying a standard distance measure between the resulting vectors. This approach may not always be able to capture the relevant notion of similarity. For example, for the “identity” feature extraction, one possibility is to take the intersection of base-pairs covered by two tracks that are compared, divided by the union of base-pairs covered by these tracks. This calculation incorporates the normalization as part of the similarity measure.

### Three canonical cases in the biological domain

The above discussion of feature extraction and similarity measures can be summarized as three different canonical analytical approaches to clustering of genomic tracks. The distinction between these three cases represent distinct notions of similarity, and thus distinct questions related to the similarity between tracks:

- **Direct sequence-level similarity** which defines similarity based on normalized coverage correspondence at the individual base pair resolution. This type of similarity can be used to answer questions regarding which tracks tend to occur at the exact same base pair positions along the genome.
- **Similarity of positional distribution along the genome** which defines similarity at a lower resolution, corresponding to similarity of smoothed versions of the genomic tracks. This is accomplished by dividing the genome into bins and comparing the normalized distribution of points/segments across these bins. This can be used to answer questions regarding which tracks display similar spectra of location preference along the genome.
- **Similarity of relations to other sets of genomic features** which defines similarity according to how points/segments of the genomic tracks to be clustered overlap with an external collection of reference tracks. This can be used to answer questions regarding which tracks display a similar preference for occurring at base pair positions associated to various functional categories. In other words, the question is not one of direct locational similarity, but of similarity of relations to other genomic features.

### Software system

Functionality for clustering of genomic tracks based on the methodology described herein is available through a Galaxy tool named ClusTrack, under the menu option “Specialized analysis of tracks”, with the submenu option “Cluster tracks based on genome level similarity” of the Genomic HyperBrowser web server [12] at URL: “http://hyperbrowser.uio.no/hb/”. This tool permits the selection of a set of genomic tracks of interest, either uploaded to the Galaxy history from local files, or selected from a large collection of tracks available from within the tool. The selected tracks can be clustered according to either of the described three canonical cases of clustering. The exact choice of feature aggregation, normalization and similarity measure, as well as the type of clustering algorithm and various parameters related to distance measure and linkage criteria, can be selected from menu lists at the web page of the tool. When selecting the “Direct sequence-level similarity” canonical case of clustering a menu is presented from which one can select versions of direct distance calculations. Similarly, for the two other canonical cases for clustering menus are presented from which specific feature aggregation methods can be selected. For “Direct sequence-level similarity” and “Similarity of positional distribution along the genome” it is then possible to in the “region&scale” section of the interface to specify the genomic region(s) that should be used for clustering. For “Similarity of positional distribution along the genome” it is in this section also possible to specify the scale, or how the selected genomic regions should be binned, for the analysis. In addition to using the graphical user interface (GUI), it is also possible to submit a batch script, specifying all input tracks and parameters, to execute any of the three canonical cases. Any clustering performed with the GUI will generate a batch script version of the same analysis and present it with the results of the run. The simplest way to to rerun a cluster analysis, but with more tracks included, is probably to modify the batch script. The batch script tool is found under the menu option “Text-based analysis interface”. Finally, the full HyperBrowser implementation, including the ClusTrack functionality, is open source and available for download from the HyperBrowser web page referred to above.

The article "ClusTrack: Feature Extraction and Similarity Measures for Clustering of Genome-Wide Data Sets" was published in 2015. Journal: PLoS One.

All three canonical cases generate dendrogram plots as output, as well as distance matrices that show the exact pairwise distances between the selected tracks. The “Similarity of positional distribution along the genome” and “Similarity of relations to other sets of genomic features” cases, which use feature matrices to calculate track distances, output these and also generate heat map plots of them with the tracks/feature vectors sorted according to calculated distances.

For the case of direct sequence-level similarity, the feature vectors are the same length as the genome, which implies a vector of for instance three billion dimensions for the human genome. Standard clustering algorithm implementations do not work with this many dimensions. We avoid the practical problem of passing such huge feature vectors into general clustering algorithms by defining suitable similarity functions that we use to compute all pairwise distances between tracks as a pre-processing step. We then pass the computed distance matrix directly to the general clustering algorithms. Note that although this works fine for most clustering algorithms, this approach cannot be used with clustering algorithms that require the computation of median feature vectors as part of the clustering process (e.g. as in k-means clustering).

### Biological example

The data clustered in the example represents occupancy data of H3K4me1 in different human cell types that were downloaded from the Roadmap of Epigenomics project [14] and ENCODE [15]. All input data used in this example are available from within the HyperBrowser server hosting the ClusTrack tool. The H3K4me1 modification was selected mainly for two reasons. The availability of data sets from many cell types and the recently described association to gene activity of H3K4me1 by its relatively high presence in the promoter of active/poised genes and in the enhancer regions of active genes [16]. Ten genomic tracks, representing H3K4me1 occupancy in five pairs of samples from immune, liver, skeletal muscle, brain and adipose cell types were selected to demonstrate the use of the GUI of ClusTrack. All the 99 available genomic tracks for H3K4me1 from within the Genomic Hyperbrowser at the time, as well as nine additional tracks of other histone modifications, were clustered to demonstrate the batch version of ClusTrack. Some of the plots generated in the demonstration of the GUI of ClusTrack is presented as figures in this paper. All analyses can be easily reproduced, and the results also accessed, by following links from the Galaxy Page [17]. The hierarchical clustering method was used, with parameters “euclidean distance” and “average” selected in the two examples were distance is not calculated directly. “Manhattan” and “maximum” distance was also tried. Hierarchical clustering allows a hierarchy of a variable number of clusters to be learned from data, suiting well our situation where we do not know what subgrouping to expect beforehand. Euclidian distance relates to the square deviation in each dimension and is widely used as a measure of similarity between feature vectors. As a measure of distance between sets of objects (subclusters), we found it reasonable to use the average of all pairwise distances between objects from each set, due to its robustness to outliers. Tracks of gene sets associated to various gene ontology (GO) terms [18], to be used as reference tracks, were created by querying the UCSC database using mySQL as a client. The query syntax is found in Supplementary Data. The query was filtered to retain only terms associated with more than 20 genes. For the batch script example, all the 383 obtained terms were used as reference tracks. For the GUI example, the number of reference tracks used was further limited to 14 by selecting only those terms with between 40 and 45 gene names associated.

The article "ClusTrack: Feature Extraction and Similarity Measures for Clustering of Genome-Wide Data Sets" was published in 2015. Journal: PLoS One.

## Results

We here introduce feature extraction approaches and similarity measures that permit genomic tracks to be clustered according to biologically relevant criteria of similarity. The approaches divide naturally into three canonical cases of clustering, where the desired similarity is based either on a) a direct correspondence of coverage at the base pair level, or b) a higher level of similarity of positional distribution, or c) similarity with respect to functional categories assigned to base pairs through an external set of reference tracks. The clustering methodology can be applied to any set of tracks defined on a common assembly version of a species. The main purpose of the methodology is to suggest subgroups within a set of tracks, which might correspond to biologically important distinctions between the entities represented by the tracks. Note that tracks that tend to overlap at the base pair level usually also follow a similar distribution across the genome. Tracks that cluster together according to case a) will therefore likely cluster together according to case b). Tracks can, however, follow a similar distribution across the genome and still not tend to overlap at the base pair level. This occurs if the tracks tend to occupy the same bins but covers different regions of the bins. Co-clustering according to case b) does, therefore, not imply co-clustering according to case a). The inherent birds eye view of distributional similarities of tracks provides support to early stages of analyses of the massive amount of data generated and continuously being released from projects like ENCODE [6].

### Clustering H3K4me1 tracks using “Direct sequence-level similarity”

The dendrogram obtained by the “Direct sequence-level similarity” case is shown in Fig 1. All sample pairs, except the one from brain, cluster together revealing that H3K4me1 tracks from samples from similar cell types overlap with each other more than they do with such tracks from other cell types. The samples from brain do, however, deviate from the rule, and cluster apart from each other, possibly reflecting that they originate from fetal and adult tissue, respectively. The dendrogram resulting from the larger number of tracks as specified in the batch script, is shown in Supplementary S1 Fig.

The article "ClusTrack: Feature Extraction and Similarity Measures for Clustering of Genome-Wide Data Sets" was published in 2015. Journal: PLoS One.

**Fig 1:** Dendrogram of H3K4me1 track clustering, using the “Direct sequence-level similarity” for the genomic region chr1-22. All samples, except the ones from brain, are placed into separate subclusters per tissue. The clustering were performed according to the canonical case “Direct sequence-level similarity”. Each individual bp-location of the genome were considered an independent feature. The distance between two feature vectors was defined as ratio of the intersection to the union of base pairs covered by two feature vectors. Clustering was performed using standard hierarchical clustering with the average linkage criterion.

### Clustering H3K4me1 tracks using “Similarity of positional distribution along the genome”

The dendrogram obtained with the “Similarity of positional distribution along the genome” case, using the relative coverage per 1 Mb bins, is shown in Fig 2. The dendrogram looks, except for having shorter branches, the same as the one resulting from “Direct sequence-level similarity”. Using “manhattan distance” did not change the structure of the dendrogram, while using “maximum distance” positioned the brain samples closer together. The dendrogram resulting from the larger number of tracks as specified in the batch script, is shown in Supplementary S2 Fig. To better appreciate the degree of co-clustering of samples of similar kind, the dendrogram of Supplementary S2 Fig was divided into subclusters based on the height of the branches. Supplementary S1 File lists these subclusters. Notably, the added fetal and adult samples do distribute to their respective sub clusters (2 and 5). Subcluster 1 contains only blood samples. Subcluster 2 contains samples from fetal or embryonic brain, including “UCSF-UBC.Fetal_Brain.HuFNSC01” from the GUI example, and also neural stem cells and two embryonic stem cell elements. Subcluster 3 is large, and is dominated by mesenchymal stem cells. Subcluster 4 contains samples from kidney, liver, muscle and adipose tissues. Subcluster 5 contains samples exclusively from adult brain. Subclusters 6 and 7 contain samples exclusively from immune cells. Subcluster 14 contains stem cells and subcluster 16 contains samples from breast.

**Fig 2:** Dendrogram of H3K4me1 track clustering using “Similarity of positional distribution along the genome” for the genomic region chr1-22. As in Fig 1, all sample pairs, except the one from brain, are placed into separate subclusters per tissue. The difference to the dendrogram of Fig 1 is only the length of branches in the dendrogram. The clustering was here performed according to the canonical case “Similarity of positional distribution along the genome”. Features were defined based on relative aggregated coverage in bins (of consecutive positions) along the genome, where the raw base pair coverage in a bin was divided by the total base pair coverage of the track across the genome (to normalize for varying overall coverage densities between tracks). Bins were defined as consecutive 1 Mbps regions along all autosomes (set in the “region&scale” section of the interface). Standard Euclidian distance was used as distance between two feature vectors. Clustering was performed using standard hierarchical clustering with the average linkage criterion.

The article "ClusTrack: Feature Extraction and Similarity Measures for Clustering of Genome-Wide Data Sets" was published in 2015. Journal: PLoS One.

### Clustering H3K4me1 tracks using “Similarity of relations to other sets of genomic features”

By using tracks representing genes associated to various gene ontology terms as reference tracks for the “Similarity of relations to other sets of genomic features” case, the H3K4me1 tracks are clustered based on functional enrichment. The dendrogram and heat map obtained when using the 14 selected reference tracks are shown in Figs 3 and 4, respectively. It can be seen that all samples from similar tissues cluster together. Changing the algorithm for calculating distance from euclidian to manhattan och maximum did not affect the structure of the dendrogram. The three reference tracks that contributed the most to the separation of the clustered tracks are “axonogenesis”, “caspase activation” and “cytokines”. Brain cells, and also liver cells to a lesser degree, have a higher H3K4me1 proportional occupancy in genes associated with the axonogenesis (nerve cell growth) term than the other cell types. Further, one can observe that genes associated with caspase activation is H3K4me1 enriched in muscle cells. This makes biological sense, since caspases are involved in apoptosis, which can be active in muscles as response to starvation and inflammation, and can be indicative of muscle differentiation [19]. Finally, genes associated with the term cytokines (immunomodulating agents, such as interleukins and interferons) are enriched by H3K4me1 in immune cells. The dendrogram of the batch script example of this case is shown in Supplementary S3 Fig. Supplementary S2 File lists the subclusters obtained by dividing the dendrogram of Supplementary S3 Fig based on the height of the branches. Fetal and adult brain samples form two subclusters just as they do in S2 Fig, but the relative distance between the two subclusters is smaller. Most of the subclusters found in Supplementary S1 File are present also in the dendrogram generated through this way of clustering. By comparing the Supplementary S1 and S2 Files, one can see that the fetal brain samples are found in subcluster 2 in both files, the mesenchymal stem cells, breast and fetal lung samples are found in subcluster 3, while the adipose tissue from subcluster 4 and the Mobilized CD34 Primary Cells from subcluster 6 in S1 File are found in subcluster 4 of S2 File. The adult brain samples are found in subclusters 5 and 8, respectively. The immune cells are found in subclusters 7 and 9, respectively. In S2 File, liver samples form their own subcluster 7. The “Similarity of relations to other sets of genomic features” generates 12 subclusters with many samples, as compared to 9 subclusters for “Similarity of positional distribution along the genome”.

The article "ClusTrack: Feature Extraction and Similarity Measures for Clustering of Genome-Wide Data Sets" was published in 2015. Journal: PLoS One.

**Fig 3:** Dendrogram of H3K4me1 track clustering using “Similarity of relations to other sets of genomic features” and 14 gene ontology reference tracks. All sample pairs were placed into separate subclusters per tissue. The separation of sample pairs into their own subclusters was stronger in this case than in Figs 1 and 2. The clustering was here performed according to the canonical case “Similarity of relations to other sets of genomic features”. Features were defined based on relative aggregated coverage (as in Fig 2) across non-consecutive sets of genome positions. Each feature was aggregated across a set of positions defined by a particular reference track. The reference tracks were again based on gene regions associated with 14 randomly selected Gene Ontology (GO) terms. Standard Euclidian distance was used as distance between two feature vectors. Clustering was performed using standard hierarchical clustering with the average linkage criterion.

**Fig 4:** Heat map plot for H3K4me1 track clustering, using “Similarity of relations to other sets of genomic features” and 14 Gene Ontology (GO) based reference tracks. The value of a specific cell in the heat map represents the relative aggregated coverage of the corresponding H3K4me1 track (as specified in the row heading) in gene regions associated with a corresponding GO term (as specified in the column heading). The rows of the heat map correspond directly to the feature vectors used to calculate the dendrogram in Fig 3.

### Follow up analysis: Functional enrichment of genes with different occupancy of H3K4me1 in fetal and adult brain

We merged the nine tracks from the adult brain subcluster 5, and the two tracks from the fetal brain subcluster 2 of Table S1, into an adult and a fetal brain track, respectively. Then, we used the Genomic HyperBrowser to find all genes for which the relative frequencies of the adult and fetal tracks were different in the body of the genes. We then extracted the Ensembl transcript IDs for these genes and submitted them to DAVID [20, 21] for functional enrichment analysis. The three top annotation clusters from a functional enrichment analysis, with terms like “pleckstrin homology” (indicating axon formation [22, 23] [24]), “neuron differentiation” and “synapse”, are listed in Table 1. The functional terms are all relevant in separating the fetal and adult brain clusters. This example illustrates how suggested subgroups not previously known or expected can direct downstream analysis, hypothesis formulation and discovery.

The article "ClusTrack: Feature Extraction and Similarity Measures for Clustering of Genome-Wide Data Sets" was published in 2015. Journal: PLoS One.

**Table 1:** Gene Ontology terms enriched by genes with different H3K4me1 occupancy in fetal and adult brain cell types.

**Category**	**Term**	**Count**	**Pop Hits**	**Benjamini**
**Annotation Cluster 1**	**Enrichment Score: 13.43**			
INTERPRO	Pleckstrin homology	88	277	3.88E-14
INTERPRO	Pleckstrin homology-type	85	303	1.83E-10
SMART	PH	88	277	1.02E-10
**Annotation Cluster 2**	**Enrichment Score: 11.59**			
GOTERM_BP_FAT	neuron projection development	76	256	1.60E-10
GOTERM_BP_FAT	neuron differentiation	109	438	1.00E-10
GOTERM_BP_FAT	axonogenesis	63	193	9.29E-11
**Annotation Cluster 3**	**Enrichment Score: 9.97**			
GOTERM_CC_FAT	synapse	99	355	1.12E-12
GOTERM_CC_FAT	cell junction	128	518	5.93E-13
SP_PIR_KEYWORDS	cell junction	101	399	1.72E-11

Table of the three top terms of the three top annotation clusters from David. The gene IDs submitted to DAVID were selected based on different H3K4me1 occupancy between fetal and adult brain clusters, by using the Genomic HyperBrowser. Benjamini = Benjamini-Hochberg.

## Discussion

As described in [9], genomic track data come in a set of intrinsically different types, and which computations are meaningful may depend on the type of track. We have here focused on the most common types of tracks: points and segments defined along the genome. Genomic data of this type may be defined as a binary vector, where every position is 1 if and only if it is covered by a point/segment. This binary vector representation formed the basis of the discussion in this manuscript. Still, the concepts introduced here, as well as most of the exact computations, can be relatively easily extended to cases of other track types. As an example, another type of track is one that assigns a numerical value to each and every base pair along the genome (denoted Function). A track of this type may for instance represent the melting propensity of DNA along the genome [25]. Two such tracks may be directly compared at the base pair level by taking the Pearson correlation of the vectors (instead of intersection divided by union, as suggested for points/segments), and their higher level similarity (or similarity of relations to other sets of genomic features) may be compared by using the mean value as aggregation (instead of a count, as suggested for points/segments).

The article "ClusTrack: Feature Extraction and Similarity Measures for Clustering of Genome-Wide Data Sets" was published in 2015. Journal: PLoS One.

A number of methods for clustering selected genomic regions based on genomic track data have been published [26–28]. This is, however, distinct from clustering multiple genomic tracks in their entirety, as described in this paper. Methods for clustering genomic regions based on data from multiple genomic tracks have also been published [28]. These methods have similarities to the recently developed methods for identifying genome chromatin states based on multiple genomic tracks defining occupancy histone modifications [29–31].

In [32], Support Vector Machines (SVM) are used to cluster ChIP-seq data from cell samples. No software is however provided. In [33], a parametric classification approach is used to infer locus specific and genome wide chromatin differences. A link to the R source code is provided.

The methods for calculating association between pairs of tracks developed in [34] have been adopted for use in clustering of ENCODE [6, 35] and ModEncode [36] data.

To give an impression of how ClusTrack can be used in various investigational scenarios, we here provide three different examples of potential ClusTrack usage (in the form of rough indications): A first example is to compare the resulting SNPs of Genome Wide Association Studies (GWAS) for various phenotypes. All three canonical cases of clustering can be relevant in this setting. Clustering the tracks using direct sequence-level similarity would represent clustering based on shared significant SNPs. Using similarity of positional distribution along the genome, with bins of for instance 1Mbp along the genome, would show similarity of location in regions corresponding roughly to regions in linkage disequilibrium. Finally, one could cluster the tracks of GWAS hits based on similarity to reference tracks of cell-type specificity (e.g. open chromatin or DHS), to see which GWAS results (set of disease associated SNPS) tend to lie in regions active in the same cell types. A second example, also involving GWAS, is to consider epigenetic data collected on GWAS cases and controls. For GWAS studies with few or no significant SNP associations it can be of interest to look for epigenetic alterations underlying the phenotypic differences between the case and control group. Clustering the case and control samples based on epigenomic data could be an introductory step to such an analysis. A third example is clustering of binding site tracks for different transcription factors (TFs), where one could look for similarity of direct binding overlap, binding in the same regions (proxy for affecting the same genes), or binding in regions active in the same cell types. Tracks of various epigenetic marks can be clustered similarly, where binding in the same regions would imply involvement in the same genomic processes.

The article "ClusTrack: Feature Extraction and Similarity Measures for Clustering of Genome-Wide Data Sets" was published in 2015. Journal: PLoS One.

## Conclusion

The approaches to feature extraction and similarity definition introduced here can serve to guide any analysis involving clustering of genomic tracks. The methodology is supported by an implementation in the form of a web tool that allows a range of fine-tuned clustering analyses to be performed on genomic data through simple choices using a set of selection boxes or through batch scripts. We demonstrate three canonical cases of clustering by applying them to tracks representing the same functional aspect from a number of different cell types. Since the results of all the three canonical cases of clustering performed in this study are generally in accordance with expectations from cell type and state information, we conclude that clustering reflects at least one aspect of the “true” track relatedness.

## Supporting Information

S1 Fig Dendrogram of H3K4me1 track clustering, using the “Direct sequence-level similarity” for the genomic region chr1-22. The dendrogram resulting from the larger number of tracks as specified in the batch script.
(EPS)

S2 Fig Dendrogram of H3K4me1 track clustering using “Similarity of positional distribution along the genome” for the genomic region chr1-22. The dendrogram resulting from the larger number of tracks as specified in the batch script. The table of S1 File lists the resulting sublclusters when this dendrogram in this figure is divided into subclusters based on the height of the branches.
(EPS)

S3 Fig Dendrogram of H3K4me1 track clustering using “Similarity of relations to other sets of genomic features” and 14 gene ontology reference tracks. The dendrogram resulting from the larger number of tracks as specified in the batch script. The table of S2 File lists the resulting sublclusters when this dendrogram in this figure is divided into subclusters based on the height of the branches.
(EPS)

S1 File Table/Excel file of subclusters for genomewide “Similarity of positional distribution along the genome”. Supplementary S2 Fig was divided into subclusters based on the height of the branches.
(XLSX)

S2 File Table/Excel file of subclusters for genomewide “Similarity of relations to other sets of genomic features”. Supplementary S3 Fig was divided into subclusters based on the height of the branches.
(XLSX)

S3 File SQL-syntax. The SQL syntax that was used in MySQL when creating the reference tracks used for the “Similarity of relations to other sets of genomic features” clustering case. The set of coordinates of genes associated to various gene ontology terms was extracted from the UCSC genome browser database.
(TXT)
